# Design of Service Robot Based on User Emotion Recognition and Environmental Monitoring

This article has been retracted.

**DOI:** 10.1155/2022/3517995

**Published:** 2022-10-04

**Authors:** Dongxu Yang

**Affiliations:** ^1^Department of Product Design, School of Art and Design, Henan University of Urban Construction, Pingdingshan 467036, China; ^2^Department of Industrial Design, Graduate School, Keimyung University, Daegu 704-701, Republic of Korea

## Abstract

Robots may be able to comprehend human emotions better by adding speech emotion recognition and environment monitoring functions to human-computer interaction systems. Robots can offer more humanized services by adapting to human emotions, resulting in a comfortable and cordial interaction between humans and robots. Improve the environment for communication and computer-human interaction and also interactive computer experience. In order for service robots to perform fluid human-computer interaction, this paper designs a sentiment analysis model based on CNN (convective neural network) to detect the feeling of interacting objects. It also builds a sentiment analysis model and an open domain dialogue system suitable for service robots. Examine the emotions experienced by the objects while they conversed. According to test results, the sentiment classification method used in this article performs more accurately on the dataset than the conventional model, and the final sentiment analysis model's F1 value can reach 0.931, which is better able to identify an emotional state. Using all voice samples as the input content of the network would eliminate the confusion between neutral emotions and other nonneutral emotions, boosting the accuracy of sentiment analysis in comparison to the fixed-length processing method of dividing or filling samples.

## 1. Introduction

Due to the continuous progress of robot industry, more and more intelligent robots appear in our lives. Robots do not only play an important role in traditional industries, medicine, agriculture, construction, and even military fields [1]. For service robots, having complete human-computer interaction ability is the premise for them to realize medical care, intelligent customer service, knowledge education, and other functional services. Service robots can be used as the intelligent auxiliary equipment for family life and the hub of the smart home. They can solve daily tasks like accompanying the elderly, accompanying children, providing domestic service, and ensuring safety, effectively reducing the pressure on young people to survive, improving the quality of life for the elderly, and enhancing the enjoyment of life for children [2]. Understanding the sensation of the interactive item is a crucial component of contemporary human-computer interaction. Applying voice emotion recognition to the human-computer interaction system can make robots have “emotion” like human beings, perceive each other's mood changes through hearing, communicate with human beings more naturally and intelligently, and endow the new human-computer interaction system with a humanized, natural, and intelligent interaction mode [3].

Service robots should be able to communicate with people on a daily basis, understand people's emotions, and make corresponding natural responses; that is, service robots should be able to listen, speak, write and know, and even understand people's thoughts and serve them [4]. The recognition system based on voice emotion can provide more novel development ideas for medical treatment, machinery, education, and service industries, further enrich people's daily life, become human helpers, and efficiently help people solve practical problems. The ability to understand emotions has become the key factor to measure whether a robot has intelligence. Service robots cannot perform the complex, and repetitive are tasks needed for machine intelligence with their basic, repetitive job. Service robots must be better equipped to recognize and interpret human emotions in order to achieve the natural interaction between man and machine. Knowing each other's current emotional states during daily interaction is the essence of human emotional intelligence. As a result, the fundamental purpose of service robots with emotional intelligence should also be the recognition of human emotional state. This paper combines CNN technology [5, 6] to create a service robot dialogue system, emotion analysis of the interactive objects in the dialogue, and an open-domain dialogue system appropriate for the service robot. This allows the service robot to conduct smooth human-computer interaction and emotion analysis of the interactive objects in the dialogue process.

With the arrival of robot industrialization era and the progress of robot technology, service robot is becoming an indispensable part of robot industry, and its development plays an important role in China's economic and social development [7]. User emotion recognition is a process that, on the basis of analyzing the changing rules of human speech signals in different emotional states, the computer can accurately extract emotional characteristic parameters that can effectively distinguish different emotions from speech messages, and the speaker's emotional states can be judged by the differences of characteristic parameters of different emotions. The user emotion recognition system can make service robots help humans to complete some specific service functions, solve many practical problems that people encounter in their lives, bring great convenience to people's lives, and improve people's happiness in life [8].

In this paper, a feature extraction method for robot speech signal recognition is proposed. CNN is used for emotion recognition, which improves the recognition accuracy of the whole system. Its main innovations and contributions are as follows: (1) in this paper, speech signals are converted into spectrograms, normalized, input to CNN, extracted speech signals features, and then classified. (2) This paper explores the emotional behaviors of different robots in perceptual situations, aiming at the emotional behaviors of robots that have an impact on users' emotional experience in perceptual situations, and explores whether they can further enhance users' emotional experience in music interaction situations, so as to clarify the impact of robot emotional behaviors on users' emotional experience in the process of music interaction.

## 2. Related Work

Following the trend of the times, service robots with voice as the main interactive mode have entered thousands of households. Moreover, with the deepening of the new generation of human-computer interaction technology and the increasing demand for emotional intelligence of service robots, the application of voice emotion recognition in service robots has gradually become a research hotspot.

With Chinese audio information and pinyin as sentiment analysis features, Kim and Park developed the reinforcement learning framework DISA based on CNN and LSTM and produced positive results [9]. In order to overcome CNN's shortcoming in long-distance context capture, Zhang merged the concepts of RNN and CNN and presented recurrent CNN for text categorization [10]. Yang et al. selected a prosodic feature set composed of statistical features such as the mean and variance of speech signal features such as energy and fundamental frequency and achieved excellent recognition rates in a multilingual emotional corpus [11]. Schuller and Schuller extracted frequency perturbations and amplitude perturbations in speech as emotion features and used hidden Markov models to perform speaker-independent emotion recognition on the SUSAS database [12]. Cui et al. utilize convolutional networks to learn from character sources, i.e., instead of using pretrained word vectors, the input is converted to character level [13]. Yan et al. found that there are differences between speech in anger, fear, and sadness, and it is reflected in the aspects of articulation intelligibility, pitch contour, average power spectrum, etc. [14]. Di and Wu used a Gaussian mixture model optimized by a kurtosis model-based selection strategy for sentiment classification [15]. Wang et al. proposed a method using fuzzy entropy to measure the effectiveness of emotion parameters combined with fuzzy comprehensive discrimination and achieved good emotion recognition results [16]. Jain et al. proposed a local feature optimization method based on cluster analysis to remove speech frames with insignificant emotional features, and the accuracy of emotion recognition was significantly improved [17]. Mohanty and Palo directly use raw audio samples to train an RNN for dimensional sentiment prediction [18].

At present, the research of speech signal recognition has made a lot of progress, but it is still one of the main problems to establish a reasonable and efficient speech signal recognition network model. In the past, there were few researches on the design of service robots based on user emotion recognition, and the recognition accuracy of emotion recognition was not high. In this paper, the scene classification of the service robot dialogue system is carried out, the speech signal recognition model of service robot is constructed by using CNN, and the word vector technology is combined to improve the recognition accuracy of the whole system.

## 3. Emotion Analysis Model of Service Robot

### 3.1. Service Robot

The central computer plays a role in the intelligent robot, and this computer has direct contact with the person who operates it [19]. Service robots work in different working environments and need different types of mobile mechanisms and working mechanisms. The actuator and driving mechanism of robot will develop towards miniaturization and integration. In the service robot, the development and use of various new vision systems and sensor devices as well as the processing and fusion of multiple sensor information are the key points for the service robot to obtain more accurate and complete environmental information and improve the intelligent decision-making level of the system. Since the service robot serves as a service, people naturally need more convenient and more natural ways to interact with the robot, including high-level emotional interaction and low-level interaction of force and touch. For all kinds of practical service robots, how to improve their adaptability to changing environment and various tasks, and improve their autonomous service ability, is a key technology with platform. According to the hierarchical architecture of AI and the overall architecture of the experimental platform, this paper analyzes the technical constraints, sets related to technical constraints for the service robot dialogue system, then analyzes the requirements of the service robot dialogue system, and puts forward the core requirements of the sentiment analysis system in this paper.

### 3.2. User Emotion Recognition

Emotional signal is a special kind of signal with its unique characteristics, such as pitch frequency, short-time zero-crossing rate, and Mel cepstrum coefficient, [20]. By recording and analyzing the emotional state of interactive objects in human-computer interaction, the real interactive experience of interactive objects can be obtained, which can be used to guide the design of the robot interactive system. According to the authenticity requirement of corpus, the topic of corpus should involve all aspects mentioned in daily communication as much as possible. The number of speakers, the gender of speakers, the age of speakers, the differences in pronunciation of Putonghua caused by different geographical locations, and the emotional state in which speakers speak, etc. all belong to the scope of the corpus. In order to ensure the authenticity of the corpus to a great extent, when building the corpus, speakers of different genders and ages should be used to collect the corpus in different emotional states.

In the research of speech signal recognition, feature selection refers to selecting a feature subset from speech signals features, and the recognition rate of speech signal recognition with this feature subset is not lower than that with the original feature set. The efficient classification model can accurately classify the speech to be tested; so, the selection of classification model is the key of speech signals recognition. The framework of the speech signal recognition system is shown in Figure 1.

Although the speech signal is fundamentally a time-varying nonstationary signal, it is known from its mechanism that inertial motion causes vocal organs to change states far more slowly than sound waves do. A frame is a segment, and the length of a frame is referred to as the frame length. Although there may or may not be overlap between frames, the continuous overlap method—in which there is overlap between subsequent frames—is typically employed for segmentation in order to guarantee the continuity and smoothness of the voice signal. Preemphasizing the voice signal is important in order to make the spectrum of the signal flatter and more equally spread from low frequency to high frequency. This makes it easier to assess spectrum and channel parameters because the same signal-to-noise ratio may be utilized in the spectrum computation. Preemphasizing the voice signal typically involves a first-order digital filter, and its expression is as follows:

(1) $$\begin{array}{c} H\left(z\right)=1-\mu z^{-1}. \end{array}$$

The preemphasis coefficient is represented by *μ*. The preemphasized speech signal has the following expression:

(2) $$\begin{array}{c} Y\left(n\right)=X\left(n\right)-\mu *X\left(n-1\right), \end{array}$$

where *Y*(*n*) represents the speech signal obtained after preemphasis, and *X*(*n*) represents the sampling value of the speech signal at *n* time. For a long time, the speech signal is unstable, but the characteristics of the speech signal are still very stable in a short time; so, we frame the speech signal.

To create a windowed speech signal *s*_*w*_(*n*), multiply the original speech signal *s*(*n*) by a movable window function *w*(*n*) with a finite window length.

(3) $$\begin{array}{c} s_{w}\left(n\right)=s\left(n\right)*w\left(n\right). \end{array}$$

By windowing voice signals, spectrum leakage brought on by framing can be avoided. Hamming window and rectangle window are the two most often used window functions. Their function expressions are as follows (the frame length is denoted by *n*):

Rectangular window:

(4) $$\begin{array}{c} w\left(n\right)=\left\{\begin{array}{c} 1,0\leq n\leq \left(N-1\right),\\ 0,n=\text{else}. \end{array}\right. \end{array}$$

Hamming window:

(5) $$\begin{array}{c} w\left(n\right)=\left\{\begin{array}{c} 0.54-0.46\cos\left[\frac{2\pi n}{\left(N-1\right)}\right],0\leq n\leq \left(N-1\right),\\ 0,n=\text{else}. \end{array}\right. \end{array}$$

Choosing the appropriate window function can make the short-term parameters better reflect the characteristics of speech signals and reduce the influence of window function on the analysis parameters of short-term signals.

For different types of questions, the corresponding replies have certain rules and strategies. The ultimate goal of scene distribution is to correctly distribute the questions in the dialogue system to the corresponding categories according to different topics. Robot speech recognition technology converts input sentences into language, but the computer directly recognizes and executes only machine language, which is not the language that humans usually speak. Speech emotion features are the basis of speech signals recognition for service robots. Whether the speech signal features extracted from the original speech signal samples are distinctive directly affects the final recognition rate of speech signals. Before speech signal feature extraction and emotion recognition, speech preprocessing is usually needed to obtain high-quality and stable speech signals. After preprocessing, the speech signal has a unified data format, and the data quality is higher, which reduces the complexity of feature analysis and extraction, and lays a good foundation for subsequent sentiment analysis.

### 3.3. User Emotion Recognition Based on CNN

A great quantity of service robots move in the indoor environment through autonomous mobile mechanisms. Because of their different service functions, they need to be equipped with different auxiliary mechanisms on the mobile platform. Autonomous mobile robots can usually be used as the basic platform of a considerable class of service robots [21]. The dialogue system requires high real-time interaction, and the system should respond as soon as possible when users use it. Real-time interaction can increase users' stickiness and experience; so, the system needs sufficient hardware support, which is mainly used for calculation. Traditional ML (machine learning) methods have made great progress in speech signal recognition. However, it is uncertain whether artificially designed feature sets can fully and effectively express emotion features. These artificially designed features depend heavily on the database, have low generalization ability, and take too long to extract features. Emotion recognition of speech is generally carried out on the speech database, and the effect of speech signal recognition is closely related to the quality of the speech database.

CNN is also often used for natural language tasks. A new matrix is generated by convolution operation between CNN convolution kernel and input matrix. Its sparse interaction is reflected in that the size of convolution kernel is much smaller than that of input matrix, because the effective features in input matrix are only a small part. Using a smaller kernel to detect features not only reduces the storage requirements of the model but also reduces the amount of computation. Because the parameters of convolution kernel are shared, convolution is superior to traditional dense matrix calculation in terms of storage requirements and statistical efficiency. Usually, in the structural design of NN (neural network), there is always a pool layer after the convolution layer. The emotional text classification based on CNN is shown in Figure 2.

When the batch normalization layer is used, the network can adopt a higher learning rate and weaken the influence of initialization parameters on network training. At the same time, the batch normalization layer also has a certain regularization property, which can reduce the dependence of the network on drop out. The essence of batch normalization layer is to normalize the layer input:

(6) $$\begin{array}{c} \hat{x}=\frac{x-\mu }{\sigma },\\ y=\gamma \hat{x}+\beta , \end{array}$$

where *x* is the input of the batch normalization layer, and *y* is the output of the normalization layer. *μ* is the mean value of *x* in the current training batch, *σ* is the standard deviation of *x* in the current training batch, *γ* is used for scaling normalized $\hat{x}$, and *β* is used for translation. The size of *μ* and *σ* depends on the training data.

When classifying texts, there are frequently clear category features present in the samples, such as particular phrases and phrases. The word embedding layer, convolution layer, pooling layer, and full connection layer are roughly combined in the CNN model for text categorization. We must create the appropriate mathematical model in accordance with the speech signals if we wish to use computers to analyze and process the emotional content of speech signals. Despite being a nonstationary random process, voice signal's properties will evolve with time. It is crucial that the service robot accurately interprets the user's input in the dialogue system. The initial step in technical processing is to understand the input intention. It can only proceed with the succeeding operation and obtain a reasonable response by evaluating the scene of the user's input statement. The pattern recognition problem of speech recognition can be investigated using ML or DL (deep learning) theory. As seen in Figure 3, the training step and prediction stage are typically included in a mainstream system structure for speech signal detection.

In the training stage, the audio samples should be subjected to corresponding preprocessing operations such as framing and windowing, and then feature extraction is performed to obtain feature vectors, which are input to the classifier for iterative training to obtain the optimal model parameters. In the prediction stage, the model parameters obtained by training are used for prediction and classification.

Suppose it is a convolution layer input sequence:

(7) $$\begin{array}{c} S=\left[x_{1},x_{2},\cdots ,x_{V},x_{T}\right]. \end{array}$$

Effective part:

(8) $$\begin{array}{c} S1=\left[x_{1},x_{2},\cdots ,x_{V}\right]. \end{array}$$

Filled part:

(9) $$\begin{array}{c} S2=\left[x_{V+1},x_{V+2},\cdots ,x_{T}\right]. \end{array}$$

Firstly, the output of *S*1 is reserved, and the output of *S*2 is ignored by element multiplication between convolution layer output Conv(*S*) and masking matrix Mask(*S*). The formula is described as follows:

(10) $$\begin{array}{c} S_{\text{conv}}=\text{Conv}\left(S\right)\times \text{Mask}\left(S\right). \end{array}$$

Let the output sequence with the same length as the input sequence *S* be

(11) $$\begin{array}{c} S_{\text{conv}}=\left[y_{1},y_{2},\cdots y_{v},\cdots y_{T}\right]. \end{array}$$

User emotion recognition is a process that, on the basis of analyzing the changing rules of human speech signals in different emotional states, the computer can accurately extract emotional characteristic parameters that can effectively distinguish different emotions from speech messages, and the speaker's emotional states can be judged by the differences of characteristic parameters of different emotions. Generally, the emotional information in voice samples is unevenly distributed among frames, with nonemotional segments and emotional segments and emotional segments with obvious and unobvious emotions. Learning all the speech frame information will cause the recognition performance of the model to decline. Therefore, it is unreasonable to assign only one emotional tag to the emotional speech sequence. It is necessary to carry out frame-level emotional tagging on the speech signal to obtain the emotional tag sequence and learn it frame by frame.

## 4. Result Analysis and Discussion

Human speech contains not only a great quantity of written symbols but also a wealth of nonverbal information such as human emotions and emotions. Traditional speech processing systems only focus on the accuracy of vocabulary information but ignore the emotional information. Voice emotion refers to the emotional information of the speaker contained in the voice signal, in which the speaker includes natural persons and computers with emotional ability. The calculation related to voice emotion is called voice emotion calculation. It calculates the emotion through the measurement, decomposition, analysis, and synthesis of speech signals, so as to automatically identify the speaker's current emotional state from his or her voice.

In the classification and recognition of some large data sets, the learning algorithm may not be able to complete the efficient recognition work until the features with poor correlation or even redundancy are removed. Therefore, reducing the number of redundant features and poor correlation with classification problems will effectively reduce the operation time of the learning algorithm and may even improve the recognition performance. Feature selection is put forward to solve this problem, which is to select a feature subset with the strongest correlation and the least redundancy from the original feature set, so as to make pattern recognition more efficient. In order to obtain high-quality dialogue, the robot question-and-answer record pairs are used as data sets, and the multi-index model based on attention is used to clean the data after 20 rounds of iterative training in DPF framework. The fitting curves of the first training loss and the last training loss of the model are shown in Figures 4 and 5, respectively.

It can be seen that in the first training, when the Epoch reaches 5.0, the loss curve of the model tends to be flat. After 20 rounds of iterative training, when Epoch reaches 3.0, the model loss can reach a stable level. Finally, the model is used to predict all the corpus, and the clean dialogue data in the whole corpus is obtained by setting the threshold. By predicting the whole corpus, we can retrieve some sentences with high quality that were deleted during the iteration of the model. The fitting curves of the first training accuracy and the last training accuracy of the model are shown in Figures 6 and 7.

It is clear that as the model's iteration times increase, the scale of the training set gets cleaner, and the model's degree of fitting likewise rises. The accuracy of the training model test set in the initial training is 0.645. The model's final test accuracy increased to 0.978 in the 20th training. In order to build CNN that satisfies the requirements, the fundamental speech signal characteristics are extracted, and the emotional speech signals are preprocessed. To train the network, the preprocessed data is fed into the created CNN. The remaining data were utilized as test sets, and 800 groups were randomly chosen as training sets. Consider the final test result of this paper to be the average value of several experiments. The results of feature recognition are shown in Table 1.

When solving the problem of pattern classification, we often want to use as many features as possible to better represent different categories, so that samples of different categories can be identified more accurately. In fact, when we combine several candidate features into one feature vector, the recognition performance is often not improved, and sometimes, the recognition performance may even drop sharply. This is because many candidate features often contain a great quantity of features with poor correlation or even redundancy with classification problems.  Table 2 is the confusion matrix of three expressions and neutrality. It can be seen from the table that the recognition rate of anger is the highest. The extracted basic features are very useful for angry judgment.

If the selected features have little discrimination ability for different categories, it is obvious that the performance of the designed classifier will be poor. Therefore, it is necessary to select features in the process of pattern recognition. Emotion recognition is a typical pattern recognition problem.  Figure 8 shows the F1 curve of different algorithms.

The test results demonstrate that the sentiment classification algorithm in this work performs more accurately on the data set when compared to the conventional model, and the final emotion analysis model's F1 value may reach 0.931, which is better able to identify the emotion state. When comparing the time domain and frequency domain recognition effects, it can be shown that the recognition effect following fusion has greatly improved. The test results clearly demonstrate the good complementarity between time domain and frequency domain characteristics, which are features derived from two different angles. The approach based on CNN provides a stronger recognition effect than the current algorithms.

## 5. Conclusion

In communication with people, language is one of the most direct and convenient ways, which reflects the emotional color of communication with people. More and more people also expect to have emotional communication with robots, hoping that robots can judge their emotional colors and output emotional expressions according to human voice, which makes the communication more humanized. The test results demonstrate that the sentiment classification algorithm in this work performs more accurately on the data set when compared to the conventional model, and the final emotion analysis model's F1 value may reach 0.931, which is better able to identify the emotion state. When comparing the time domain and frequency domain recognition effects, it can be shown that the recognition effect following fusion has greatly improved. The test results clearly demonstrate the good complementarity between time domain and frequency domain characteristics, which are features derived from two different angles. The approach based on CNN provides a stronger recognition effect than the current algorithms. The depth features extracted by this algorithm are the deep features of voice emotion extracted from two aspects, which can learn voice emotion signals from time domain and frequency domain, and retain the original information of voice emotion well. At present, there are few open-source Chinese corpora, and the training of DL models needs a lot of high-quality data. Therefore, it is necessary to collect dialogue data in the subsequent use process, build a large corpus, and dynamically optimize the dialogue system to generate models.

## Figures and Tables

**Figure 1:** User emotion recognition system framework.

**Figure 2:** CNN is used for speech signal text classification.

**Figure 3:** User emotion recognition process based on DL.

**Figure 4:** First training loss curve.

**Figure 5:** Loss curve of 20th training session.

**Figure 6:** Accuracy curve of the first training.

**Figure 7:** Accuracy curve of 20th training.

**Figure 8:** F1 curve of different algorithms.

**Table 1:** Correct rate of speech signal recognition based on CNN.

Characteristic	Discrimination
ZCR	76.5
Amplitude	78.2
Energy	78.3
ZCR+ amplitude+ energy	75.9
Energy+ZCR	82.2
Amplitude+ energy	77.8
ZCR+ amplitude	80.3

**Table 2:** Confusion matrix of three emotions.

	Happy	Sad	Angry
Happy	86	14	0
Sad	28	82	0
Angry	0	0	100

## Data Availability

The data used to support the findings of this study are available from the corresponding author upon request.
